This article has been retracted.

# The RPL4P4 Pseudogene Is a Prognostic Biomarker and Is Associated with Immune Infiltration in Glioma

**DOI:** 10.1155/2022/7967722

**Published:** 2022-08-09

**Authors:** Zengliang Wang, Yirizhati Aili, Yongxin Wang, Nuersimanguli Maimaitiming, Hu Qin, Wenyu Ji, Guofeng Fan, Bo Li

**Affiliations:** ^1^Department of Neurosurgery, Xinjiang Bazhou People's Hospital, Xinjiang, China; ^2^Department of Neurosurgery, First Affiliated Hospital of Xinjiang Medical University, Urumqi, Xinjiang, China; ^3^Department of Oncology, First Affiliated Hospital of Xinjiang Medical University, Urumqi, Xinjiang, China; ^4^Department of Neurosurgery, Affiliated Hospital of Jining Medical University, Jining, Shandong, China

## Abstract

**Objective:**

Research over the past decade has suggested important roles for pseudogenes in gliomas. Our previous study found that the RPL4P4 pseudogene is highly expressed in gliomas. However, its biological function in gliomas remains unclear.

**Methods:**

In this study, we analyzed clinical data on patients with glioma obtained from The Cancer Genome Atlas (TCGA), the Chinese Glioma Genome Atlas (CGGA), the Genotype-Tissue Expression (GTEx), and the GEPIA2 databases. We used the R language for the main analysis. Correlations among RPL4P4 expression, pathological characteristics, clinical outcome, and biological function were evaluated. In addition, the correlations of RPL4P4 expression with immune cell infiltration and glioma progression were analyzed. Finally, wound healing, Transwell, and CCK-8 assays were performed to analyze the function of RPL4P4 in glioma cells.

**Result:**

We found that RPL4P4 is highly expressed in glioma tissues and is associated with poor prognosis, IDH1 wild type, codeletion of 1p19q, and age. Multivariate analysis and the nomogram model showed that high RPL4P4 expression was an independent risk factor for glioma prognosis and had better prognostic prediction power. Moreover, high RPL4P4 expression correlated with immune cell infiltration, which showed a significant positive association with M2-type macrophages. Finally, RPL4P4 knockdown in glioma cell lines caused decreased glioma cell proliferation, invasion, and migration capacity.

**Conclusion:**

Our data suggest that RPL4P4 can function as an independent prognostic predictor of glioma. It also shows that RPL4P4 expression correlates with immune cell infiltration and that targeting RPL4P4 may be a new strategy for the treatment of glioma patients.

## 1. Introduction

Gliomas are common primary brain tumors characterized by treatment resistance, high recurrence, and high mortality rates. Gliomas have been classified into four grades, with grades III and IV usually leading to poor clinical outcomes [1]. Lower-grade gliomas (LGGs) can progress to higher-grade gliomas (GBM, for glioblastoma multiforme), which are resistant to chemotherapy. Despite various treatment modalities, including surgical intervention, postoperative adjuvant chemoradiotherapy, and immunotherapy, patients with gliomas exhibit poor prognoses [2]. In recent years, with the development of molecular pathology, some molecular markers in glioma have played an important role in the diagnosis and prognosis of the disease. These molecular markers include isocitrate dehydrogenase (IDH), epidermal growth factor receptor (EGFR), O-6-methylguanine-DNA methyltransferase (MGMT), and tumor protein p53 (TP53) [3]. In 2021, the WHO CNS5 placed even more emphasis on the importance of molecular markers in glioma [4]. Therefore, the new molecular classification of glioma may play a key role in its prognosis.

Pseudogenes are a class of homologous genes similar to functional genes and are unable to express truly functional proteins due to mutations in their coding sequence (such as insertion, deletion, and code shift mutations) and to the premature appearance of stop codons [5]. For a long time since its discovery, pseudogenes have been thought to be nonfunctional, “junk genes” and “fossil genes”, but some recent studies have found that some pseudogenes have certain functions, can be transcribed, and can also be regulated in other ways to encode DNA function [6]. Pseudogenes may be associated with a variety of cancers and may function as oncogenes or tumor suppressor genes involved in the development of certain cancers [7]. Pseudogenes have a variety of functions, serving as bait for mRNA and proteins and acting as competitive endogenous RNAs for microRNA sponges. There are endogenous interfering RNAs with pseudogene production, and interference mechanisms for RNA can be formed in subsequent development [8]. The pseudogene itself and the endogenous small interfering RNAs it produces can have a regulatory effect on their parent genes after transcription [9]. The significance of pseudogenes in gliomas has rarely been studied, and there are no systematic studies on prognosis-related pseudogenes and on the role of pseudogenes in the malignant evolution of gliomas.

Mutations in ribosome proteins, ribosomal RNA (rRNA) processing, and ribosome assembly factors can lead to ribosome disease, which is associated with an increased risk of developing malignancy [10]. Recent studies link ribosome protein mutations and abnormal ribosomes to poor prognosis, highlighting that ribosome protein targeted therapy is a promising treatment for cancer patients [11]. Ribosomal protein genes have the largest number of processed pseudogenes, approximately 1700; these genes include cyclophilin A, actin, keratin (keratin), GAPDH, cytochrome C (cytochrome C), and nucleophosmin [12]. There are many copies of the processed pseudogenes. Hirotsune et al. [13] found that pathological changes occur when the function of the ribosomal protein pseudogene in mice is blocked. Therefore, it has been theoretically asserted that the functional abnormalities of pseudogenes may be related to the occurrence of multiple diseases. Ribosomal protein L4 pseudogene 4 (RPL4P4) belongs to the ribosomal protein pseudogene that plays a regulatory role in protein folding and protein posttranslational modification [14]. Studies have shown that RPL4P4 is closely related to the maintenance of normal human function, and its loss of expression is associated with tumors, endocrine dysfunction, and immune diseases [15]. In our previous studies, we found that the differential expression of RPL4P4 is associated with the occurrence and development of multiple tumors (DLBC, GBM, LGG, TGCT, and THYM). Among them, there is a clear correlation with glioma, and the pattern of RPL4P4 expression, its prognostic value, and its correlation with the tumor microenvironment in glioma remain unclear.

To further understand the potential role of RPL4P4 in glioma, this study investigated the diagnostic and prognostic significance of RPL4P4 in glioma by data mining datasets from TCGA, GTEx, and CGGA. Subsequently, GO, KEGG, and GSEA analyses were used to determine the possible biological functions and mechanisms of RPL4P4 in glioma. In addition, the relationship between RPL4P4 expression and the infiltration of immune cells in glioma was assessed in the Tumor Immune Estimation Resource (TIMER) database. Finally, we investigated the effects of RPL4P4 on the biological behavior of glioma cell lines in a variety of ways. These findings indicate that RPL4P4 can regulate the infiltration of immune cells into gliomas and that the level of RPL4P4 expression may be a prognostic biomarker in patients with these tumors.

## 2. Materials and Methods

### 2.1. Microarray Data Information

The data used in our study were obtained from the public databases The Cancer Genome Atlas (TCGA, https://tcga-data.nci.nih.gov/tcga/), Genotype-Tissue Expression (GTEx, https://www.gtexportal.org), and Chinese Glioma Genome Atlas (CGGA, http://www.cgga.org.cn.). TCGA and GTEx data were used as the experimental groups, and CGGA data were used as the validation set. The expression data of TCGA glioma, including TCGA lower-grade tissues (LGG) and TCGA high-grade glioma tissues (GBM), were downloaded from the TCGA database. The dataset consisted of the clinical data of 698 glioma patients and 5 normal individuals, and patients with incomplete clinical data were excluded from subsequent analyses. In addition, the validation set (CGGA data), gene expression data, and corresponding clinical data of the glioma patients were downloaded from CGGA (LGG+GBM). Two datasets containing the clinical data of 693 and 325 patients (mRNAseq-693 and mRNAseq-325), respectively, were downloaded. The two sets of gene expression data were corrected in batches and integrated by loading them into the Limma and SVA packages in R software (v 4.1.2). The prognostic value of RPL4P4 expression in various cancers was analyzed using the GEPIA2 [16] database.

### 2.2. Difference and Survival Analyses

Transcription data from TCGA and GTEx datasets were integrated, and RPL4P4 transcription data were selected. Then, the expression levels were compared between the tumor and normal groups. After integrating RPL4P4 expression with clinical data, we divided the data into high and low expression groups based on the medium level. Next, we performed survival analyses among the TCGA, GTEx, and CGGA datasets.

### 2.3. Clinical Analyses

Since clinical data in the TGGA database were the most comprehensive and the data volume was sufficient, conclusions drawn from it have the highest reliability. The main clinical characteristics were as follows: age, sex, chemoradiotherapy status, WHO grade, histological type, critical molecular pathology information, and survival data. Univariate and multivariate analyses were performed to explore clinical factors associated with prognosis. Subsequently, associations between RPL4P4 expression levels and various clinical subgroups were observed. On this basis, the nomogram prediction model was established, visually analyzed, and evaluated by the C-index and calibration curve. The R packages “rms,” “beeswarm,” and “survivalROC” were used during this process.

### 2.4. GO Annotation and KEGG Pathway Enrichment Analysis

Gene set enrichment analysis (GSEA) is a useful tool to interpret gene expression profiles and obtain insights into biological mechanisms; it evaluates microarray data at the level of gene sets. In our study, each sample was divided into high, medium, and low expression groups based on RPL4P4 expression levels. Through Bayesian correction, we explored major enrichment pathways for various differentially expressed genes among the high- and low-expression groups and included Kyoto Encyclopedia of Genes and Genomes (KEGG) and Gene Ontology (GO) term enrichment analyses. This reminded us to give more attention to potential pathways.

### 2.5. Immune Cell Infiltration Analysis

The associations between RPL4P4 expression and glioma infiltration by B cells, CD4+ T cells, CD8+ T cells, macrophages, neutrophils, and dendritic cells were examined using the TIMER database (http://timer.cistrome.org) [17], with analyses performed using the R package GSVA.

### 2.6. Cell Line and Cell Culture

All cell lines, including U-251 and A-172, were purchased from the Cell Bank of the Chinese Academy of Sciences (China). All cell lines were cultured in DMEM with 10% newborn bovine serum supplemented with 100 U/mL penicillin and 100 *μ*g/mL streptomycin in a 5% CO_2_ incubator with saturated humidity and 37°C constant temperature.

### 2.7. Construction and Transfection of Lentivirus

The cells were cultured. When the cell growth density reached more than 85%, the original medium was aspirated and 5 mL of fresh serum-free 1640 medium was added. The culture was continued for 6 h to make the cells hungry and then prepared for cell transfection. For transfection, 40 *μ*L of lentiviral infection preparation A solution and 40 *μ*L of P solution (HitransG A infection enhancer 25× and HitransG P infection enhancement solution 25×) (gene sequence 1 5′-GCCCAATGATATCGGTGTACT-3′, gene sequence 1 2′GCAGAGCTATGGCTCGAATTC-3′, and gene sequence 1 3′GGGCCTGTGCATCATCTATAA-3′) were each added to 1.5 mL enzymatic EP tubes, followed by 5 *μ*L of viral stock solution to mix it. The solution was then inoculated in a T25-well plate at a viral MOI value of 5 (the recommended concentration in the instruction manual) and gently inverted and mixed several times. The two tubes of reagents described above were mixed and gently inverted several times. The prepared transfection reagent was slowly and evenly dripped into the Petri dish, and then, the mixture was gently shaken, placed in a constant temperature cell culture incubator at 37°C and 5% CO_2_, and cultured for 24 h after the fluorescence microscope began to detect the cell fluorescence strength and cell growth state. When the abundance of fluorescent cells was approximately 80%, the medium was replaced with complete medium added to puromycin to continue to culture and screen successfully transfected cells. Puromycin (biosharp purine mycin solution 10 mg/mL) was dissolved in complete medium to screen for 2-3 days at a concentration of 2 *μ*g/mL, after which cells were cultured with normal culture medium and passaged according to the number of cells grown. According to the Declaration of Helsinki, the samples and case data used in this study were approved by the Ethics Committee of the First Affiliated Hospital of Xinjiang Medical University.

### 2.8. Puromycin Kill Curve

Cells were spread in 6-well plates with approximately 80% confluence, added to the appropriate viral solution and polybrene (final concentration of 5-10 g/mL), and incubated in an incubator overnight. The medium containing the screening drug blasticidin/puromycin was replaced to screen for stable transformants. The medium was changed every 3 to 4 days until resistant clones appeared. At least five resistant clones were picked, the culture was expanded, and the target gene and protein expression were identified. Control was set as an empty vector.

### 2.9. Transwell Assay

Transwell cells were placed in a 24-well plate, substrate glue was added to the Transwell cells, and complete culture medium was added to the substrate. After digestion and resuspension, the cells of each group were inoculated in the upper chamber of the Transwell, and the number of cells was 3 × 10^4^. After 48 h of culture, the cells that did not invade the subchamber were washed away. Then, the cells were fixed with 4% polymethanol and stained with 0.1% crystal violet for 20 min. The number of cells invading the subcompartment in each field was counted under an inverted microscope.

### 2.10. Wound Healing Assay

The cells in each group were digested by trypsin and inoculated into 6-well plates with 1 × 10^6^ cells in each well. Then, the cells were cultured at 37°C, 5% CO_2_, and 100% relative humidity until the cells reached approximately 90% confluence. Then, cells were scratched from top to bottom with a 200 *μ*L pipette tip, and the scratched cells were washed away with PBS buffer. Then, the culture was continued for 24 h under the same conditions. The single-layer images were observed using an inverted microscope, and the migration ability of cells was analyzed by measuring the distance moved by the cell front and the width of the scratch.

### 2.11. CCK-8 Kit for Cell Value-Added Experiments

After the cell density reached approximately 90%, the cell culture was washed with PBS twice, underwent pancreatic enzyme digestion, and was then resuspended into a 15 mL centrifuge tube. According to the kit instructions, the experimental protocol was performed as follows: the cell suspension was inoculated in a 96-well plate (cell count is 5000-10,000/100 *μ*L) and then incubated at 37°C and 5% CO_2_ for 2-4 hours. Cell adherence was examined at the following times: 0 h, 6 h, 12 h, 24 h, and 36 h. Subsequently, 10 *μ*L of CCK-8 (Bioss enhanced cell counting kit-8 size: 500 T) was added to the wells for 48 h to avoid bubble production, which were then placed in the incubator for 2 h. The absorbance at 450 nm was determined with a microplate reader.

### 2.12. Statistical Analyses

Statistical analyses of the datasets from the TCGA database were performed using R (v 4.1.1) software. The associations between RPL4P4 and pathologic characteristics were evaluated by the Wilcoxon rank sum tests for continuous variables and chi-square tests for categorical variables. Overall survival (OS), disease-free survival (DFS), and progression-free interval (PFS) were calculated using the Kaplan-Meier method and compared by log-rank tests. The univariate and multivariate Cox regression analyses were performed to assess the correlation between clinical features and survival (OS and DFS). For data regarding the function of RPL4P4, statistical analyses were performed using GraphPad Prism 7.0 software. Differences between two groups were assessed using Student's *t* tests, and differences among multiple groups were evaluated by one-way ANOVA. *P* values < 0.05 were considered statistically significant.

## 3. Results

### 3.1. Expression and Prognostic Potential of RPL4P4 in Pancancer Analysis

First, we used VASH1 expression levels in cancer and normal tissue samples from the TCGGA database. Given the limited number of normal samples in the TCGGA database, we integrated the RPL4P4 expression of cancer tissue and normal tissue samples from the GTEx and TCGGA databases and found that there was a significant difference in the expression of RPL4P4 in multiple cancers compared to the normal GTEx control group (Figure 1(a)). Furthermore, through GEPIA analysis, RPL4P4 and DLBC, GBM, LGG, TGCT, and THYM were associated (Figure 1(b)), all of which suggest that they play an important role in the development of glioma. We performed a univariate analysis using the TCGA dataset. The forest plot showed that in 33 cancers, RPL4P4 had a significant effect on the survival time according to specific tumor types, and RPL4P4 had a clear correlation with prognosis in patients with gliomas (*P* < 0.001) (Supplemental Figure 1). For further exploration, we analyzed the differential expression of RPL4P4 in glioma and normal tissues using TCGA and then used the GEPIA online analysis website for the verification of the results. The results showed that RPL4P4 was highly expressed in glioma tissues (Figure 1(c)). Based on median RPL4P4 expression in samples from the databases used, patients were grouped according to their high or low levels of RPL4P4 expression. We found that high RPL4P4 expression was correlated with poorer OS (*P* < 0.001) (Figure 1(d)). We evaluated the model by the tROC curve and found that it had good specificity and sensitivity (AUC = 0.692) (Figure 1(e)).

### 3.2. RPL4P4 Expression Is Significantly Correlated with the Degree of Malignancy and Glioma Subtype

We further analyzed and visualized heatmaps of RPL4P4 and glioma clinical features in the TCGA database and found that RPL4P4 was correlated with the clinical features of glioma. Through a correlation analysis with clinical data (Table 1), we found that high RPL4P4 expression was significantly correlated with that of other WHO subtypes, IDH1 mutation status, histological types, and age (Figure 1(f)) and that RPL4P4 was significantly higher in WHO IV expression. To further confirm that we used the CGGA database, high RPL4P4 expression correlated with WHO subtypes, IDH1 mutation status, codeletion of chromosomes 1p and 19, and age (Figure 1(g)). We found that there were significant differences between the WHO grade subgroups, which were positively correlated with the malignancy of glioma (Supplemental Table 1).

### 3.3. Univariate and Multivariate Analysis Showed the Prognostic Significance of RPL4P4 and Its Association with Related Clinicopathological Factors in Glioma

Based on the median RPL4P4 expression in the samples in the database, patients were divided into groups with high and low levels of RPL4P4 expression. High RPL4P4 expression was found to correlate with poor OS (Figure 2(a)), DFS (Figure 2(b)), and PFS (Figure 2(c)), and a visual forest plot was plotted (Figures 2(d)–2(f)) (Supplemental Tables 2, 3). Univariate results showed that high RPL4P4 expression in gliomas was significantly associated with a poor prognosis (Table 2). Combined with the results of multivariate analyses, high WHO grade, PD, IDH1 wild type, high RPL4P4 expression, age, and histological type are risk factors for glioma prognosis. The above results further confirm that increased RPL4P4 expression is associated with the development of malignant glioma. The ability of a nomogram that included RPL4P4 expression, age, IDH mutation status, primary therapy outcome, 1p19q codeletion, and WHO grade to accurately predict prognosis in glioma patients was tested. This nomogram was found to predict 1-, 3-, and 5-year OS in patients with glioma (Figure 2(g)), demonstrated the accuracy of the model with a calibration curve, and found that the 1-, 3-, and 5-year models had good predictive performance (Figure 2(h)). In summary, RPL4P4 is an independent risk factor for glioma prognosis, helps to predict patient prognosis and is a potential biomarker for glioma.

### 3.4. The Prognostic Value of RPL4P4 in Different Glioma Subgroups

Assessment of the prognostic value of RPL4P4 expression in glioma patients subgrouped by WHO grade, 1p/19q codeletion, IDH mutation status, recurrence, and age showed that high expression of RPL4P4 was associated with poor prognosis in all of these groups (Figures 3(a)–3(h)). These results suggested that gliomas with high RPL4P4 expression were associated with poor outcomes in response to treatment.

### 3.5. Genes Coexpressed with RPL4P4 and Enrichment Analysis in Patients with Glioma

To further elucidate the importance of RPL4P4 in glioma, we explored the coexpression patterns of RPL4P4 using the LinkFinder module in LinkedOmics. We obtained 316 associated genes and extracted the 10 most relevant genes using the chord diagram (Figure 4(a)). A heatmap was constructed showing the 50 most significant genes positively associated with RPL4P4 expression in glioma (Figure 4(b)). Subsequently, we performed a gene function enrichment analysis, showing the enrichment results using GO and KEGG tools with bubble plots. Annotations to the GO term suggest that many genes expressed with RPL4P4 are involved in biological processes such as negative regulation of gene expression, negative regulation at the chromatin level, nucleosome formation, participation in transcriptional regulation, and humoral immune response. Molecular functional annotations of these GO terms indicate that genes coexpressed with RPL4P4 are primarily involved in negative regulatory processes, i.e., manifested as inhibition of translational and transcriptional levels, ribosomal protein activity, and immune response correlation (Figures 4(c)–4(e)). KEGG pathway enrichment suggests that genes coexpressed with RPL4P4 participate in neuroactive ligand-receptor interactions, alcoholism, neutrophil extracellular trap formation, nicotine addiction, morphine addiction, GABAergic synapses, EMC-receptor interactions, retrograde endocannabinoid signaling, and calcium signaling pathways (Figures 4(f) and 4(g)).

### 3.6. Function and Somatic Mutation of RPL4P4

GSEA tools were utilized to identify the signaling pathways involving RPL4P4 in glioma. High RPL4P4 expression was found to be involved in neurotransmitter secretion, neurotransmitter transport, potassium ion transport, regulation of neurotransmitter levels, regulation of synaptic plasticity, calcium signaling pathways, long-term potentiation, neuroactive ligand receptor interactions, phosphatidylinositol signaling pathways, and ribosomes (Figures 5(a) and 5(b)).

In addition, we obtained the driver gene for gliomas and evaluated somatic mutations in patients with RPL4P4 at different levels of expression.  Figure 5(c) shows the mutation distribution of the 15 driver genes with the highest frequency of change in the high and low RPL4P4 groups, of which the high expression of RPL4P4 and the low expression of VASH1 have a strong correlation with IDH1, and further correlation analysis shows that RPL4P4 is positively correlated with the status of IDH1 (*r* = 0.407, *P* < 0.001) (Figure 5(d)). These results suggest that RPL4P4 combined with IDH1 may have some significance for glioma risk stratification and for guiding treatment.

### 3.7. Correlation of RPL4P4 Expression with Immune Cell Infiltration and Immune Checkpoints in Glioma Patients

To display the distribution of immune infiltration in glioma, we first explored the immune infiltration of 22 subpopulations of immune cells in glioma tissue using the CIBERSORT algorithm. The divergence in tumor-infiltrating immune cells (TIICs) may be a distinctive feature of individual differences and may have prognostic value (Figures 6(a) and 6(b)).  Figure 6(a) shows that RPL4P4 expression is positively correlated with the infiltration of neutrophils, M0 and M2 macrophages, eosinophils, DCs, and Treg T cells in gliomas. It was inversely correlated with mast cell and B cell infiltrates. Next, we investigated the relationship between RPL4P4 and tumor purity based on the ESTIMATE algorithm. In gliomas, RPL4P4 expression was positively correlated with stromal score, immune score, and ESTIMATE score (Figure 6(c)). RPL4P4 was also positively correlated with tumor mutation burden (TMB) (Figure 6(d)). The above evidence suggests that RPL4P4 is a potential marker of tumor microenvironmental status.

We further confirmed the value of six types of immune-infiltrating cells in predicting LGG prognosis by TIMER (Figure 6(e)). Differential correlation analysis showed that tumor immune infiltrators were correlated with RPL4P4 in 11, of which M0 macrophages (0.4), M2 macrophages (0.23), neutrophils (0.22), CD8+ T cells (0.15), and gamma T cells were positively correlated and DC cells, eosinophils, mast cells, eosinophils, NK cells, and CD4+ T cells were negatively correlated. The above results suggest that RPL4P4 is clearly associated with M2 macrophages, which may promote the formation of an inhibitory immune microenvironment, thereby promoting tumor progression and leading to a poor prognosis (Figure 6(f)).

Given that immunotherapy is a key treatment for tumor reduction and eradication, the relationship between RPL4P4 expression and gene expression at 47 immune checkpoints was further analyzed. Interestingly, the analysis showed that RPL4P4 expression was positively correlated with the immune checkpoint gene commonly found in multiple cancers. In gliomas, RPL4P4 is closely related to the expression of CD276, NRP1, CD40 and CD48 (Figures 7(a) and 7(b)). This suggests a potential synergy between RPL4P4 and consistent immune checkpoints. The complex pattern of RPL4P4 modulating tumor immune responses by modulating immune checkpoint genes is important. In addition, we identified the relationship between RPL4P4 and TMB, microsatellite instability (MSI), and mismatch repairs (MMRs), which showed that gliomas were inversely correlated with MSI and MMRs, which further supported the above conclusions (Figures 7(c) and 7(d)).

### 3.8. RPL4P4 Knockdown Inhibits the Proliferation, Migration, and Invasion of Gliomas

To demonstrate that RPL4P4 affects glioma cells, the RPL4P4 gene was silenced by three lentiviral transfections of glioma cell lines (A-172 and U-251). By screening stable transfection lines using the puromycin kill curve, the highest transfection efficiency was found in gene sequence 1 5′-GCCCAATGATATCGGTGTACT-3′ (53.7%), so this gene sequence was selected as the lentivirus for the next experiment (Figure 8(a)). The transfected cell lines were divided into control, si-NC, and si-RPL4P4. We confirmed the proliferative effect of the RPL4P4 gene on glioma cells through the CCK-8 trial. After silencing RPL4P4 expression, the proliferation capacity of glioma cells (A-172 and U-251) in the si-RPL4P4 group decreased significantly compared with the that of other groups (Figures 8(b) and 8(c)). In addition, the cell scratch test found that the healing ability of si-RPL4P4 glioma cells was significantly lower than that of the control and si-NC groups (*P* < 0.05) (Figures 8(d) and 8(g)). Finally, we conducted a Transwell invasion test to confirm the effect of RPL4P4 on the aggressive ability of glioma cells and found that the glioma cell invasion ability of si-RPL4P4 was significantly lower than that of the control and si-NC groups (*P* < 0.05) (Figures 8(h) and 8(i)). Overall, these results suggest that RPL4P4 expression is significantly associated with the ability of glioma cells to invade, migrate, and proliferate.

## 4. Discussion

Gliomas are the most common type of primary malignant brain tumor in adults [18, 19]. They are associated with short survival and direct repercussions on quality of life and cognitive functions [20]. Even with standard therapy, including surgical resection, radiotherapy, and chemotherapy, the prognosis for glioma patients remains poor [2, 21]. Further advancements in technologies that identify new biomarkers to improve the understanding of the regulation of cell processes and treatment of glioma are needed.

In recent years, the roles of pseudogenes have been reported to be associated with various human diseases, including cancer, and have attracted much attention [22]. Several pseudogenes are differentially expressed in glioma tissues and are implicated in biological processes related to tumorigenesis and drug resistance to chemotherapy [23, 24]. To date, no report has investigated the function and mechanism of the pseudogene RPL4P4 in glioma. These findings shed new light on the importance of the orchestrated interactions among pseudogenes, microRNAs, and proteins in tumorigenesis and may be used for precision therapy in glioma patients.

To our knowledge, the present study is the first to comprehensively evaluate RPL4P4 expression and its association with clinical and prognostic outcomes in glioma using various public databases, including the CGGA, TCGA, GEPA2, and UALCAN datasets. We found that RPL4P4 was significantly overexpressed in gliomas and that increased RPL4P4 expression correlated significantly with poor outcomes, tumor grade, age, IDH mutation status, and chromosome 1p/19q codeletion status. Univariate and Cox analyses showed that RPL4P4 expression correlated positively with WHO grade, primary therapy outcome, IDH mutation status, age, and poor OS in patients with glioma. Based on the multivariate Cox analysis, a nomogram was constructed to predict the prognosis of patients with glioma based on the expression of RPL4P4 and to stratify glioma patients with better performance. Furthermore, GSEA showed that high RPL4P4 expression was positively correlated with neurotransmitter secretion, neurotransmitter transport, potassium ion transport, regulation of neurotransmitter levels, regulation of synaptic plasticity, calcium signaling pathways, long-term potentiation, neuroactive ligand receptor interaction, phosphatidylinositol signaling pathways, and ribosomes. Further inferred from the pathways involved, RPL4P4 may act as an oncogene, regulating the expression of ribosomal genes at the stage, thus promoting gliogenesis.

Immunotherapy plays an increasingly important role in standard cancer treatment, as it can recruit tumor-infiltrating T cells to eradicate tumor cells. In glioma, tumor-infiltrating CD4+ T cells play an important role in immune regulation [25, 26]. GSEA showed that RPL4P4 expression was significantly involved in immune signaling pathways. Analysis of immune cell infiltration in the present study showed that high RPL4P4 expression was significantly and positively associated with levels of M0 macrophages (0.4), M2 macrophages (0.23), neutrophils (0.22), CD8+ T cells (0.15), and gamma T cells in gliomas. Among them, M2 macrophage infiltration is clearly related, and M2-like tumor-associated macrophages play an important role in the immune microenvironment of gliomas [27], and the high expression of RPL4P4 promotes the inhibitory phenotype of macrophages, thereby promoting tumor progression, which indicates that RPL4P4 may serve as a potential biomarker. Inhibition of its expression may improve the sensitivity of gliomas to immunotherapy, and this result needs to be further confirmed.

The biological functions of RPL4P4 in these cells were evaluated by RPL4P4 knockdown, which significantly inhibited glioma cell proliferation, invasion, and migration. These results suggest that NRPL4P4 may act as an oncogene in glioma, but additional studies are needed to confirm these findings.

This study had several limitations. Although we explored the correlation between RPL4P4 and immune cell infiltration in glioma patients, we did not determine the function of RPL4P4 in regulating the tumor microenvironment in glioma. In addition, we showed that a depletion of RPL4P4 could inhibit the migration of glioma cells, but the potential molecular mechanisms of RPL4P4 in cancer metastasis remain unclear. Furthermore, the present study assessed the expression and biological roles of RPL4P4 in databases of patients with glioma and cultured cells, not in vivo. Additional studies are required to assess the function of RPL4P4 in glioma metastasis and in regulating the tumor microenvironment of glioma.

## 5. Conclusion

In summary, these findings shed new light on the importance of the pseudogene RPL4P4 in glioma. The results showed that RPL4P4 expression was increased in glioma tissues and that its high expression correlated with the malignant progression of gliomas. RPL4P4 knockdown in glioma cells reduced their proliferation and migration activities. In tumor immunity, RPL4P4 was significantly associated with M2-like tumor-associated macrophages in the microenvironment of gliomas. Therefore, RPL4P4 is a prognostic biomarker linked to immunosuppression, and targeting RPL4P4 may improve the outcome of immunotherapy.

## Figures and Tables

**Figure 1:** RPL4P4 expression and prognostic value in glioma. (a) The transcription level of RPL4P4 was determined in different tumor tissues and normal tissues by GEPIA2. (b) The mRNA expression levels of RPL4P4 in different tumor tissues and normal tissues analyzed by TCGA and GTEx. (c) RPL4P4 expression is significantly upregulated in glioma. (d) Kaplan-Meier survival analysis of all gliomas. (e) tROC analysis showing the predictive value of RPL4P4based TCGA glioma. (f) The correlation between RPL4P4 expression and different clinical features based on TCGA glioma. (g) The correlation between RPL4P4 expression and different clinical features based on CGGA. ^∗^*P* < .05, ^∗∗^*P* < .01, and ^∗∗∗^*P* < .001.

**Figure 2:** The prognostic value of RPL4P4 in glioma. (a–c) The prognosis of RPL4P4 in glioma examined by TCGA databases. (d–f) The forest plot indicates the prognosis in the presence of (d) OS, (e) DFS, and (f) PFS. (g) Construction of a nomogram to predict OS. (h) The calibration curve used to display the TCGA glioma cohort for OS.

**Figure 3:** Analysis of the prognostic value of RPL4P4 in different glioma subgroups. (a–h) Analysis of the prognostic value of RPL4P4 in different subgroups.

**Figure 4:** Analysis of the biological function of RPL4P4 in glioma. (a and b) The coexpression of the RPL4P4 gene in glioma was explored by LinkedOmics. (c–g) GO and KEGG analyses of genes coexpressed with RPL4P4 in glioma.

**Figure 5:** Function and somatic mutation of RPL4P4. (a and b) The involvement of genes coexpressed with RPL4P4 in glioma signaling pathways as examined by GSEA software. (c) Molecules associated with a somatic mutation describe RPL4P4 mutations in glioma. (d) Correlation between RPL4P4 and IDH1.

**Figure 6:** Relationship between the expression of RPL4P4 and the level of immune infiltration in glioma. (a and b) Correlation matrix for all 22 immune cell proportions. (c) Correlation between RPL4P4 and ImmuneScore, ESTIMATEScore, and StromalScore in glioma. (d) RPL4P4 expression was positively correlated with TMB. (e) The correlation between RPL4P4 expression and the infiltration of different immune cells based on time. (f) Correlation between RPL4P4 expression and immune-infiltrating cells in TCGA. ^∗^*P* < .05, ^∗∗^*P* < .01, and ^∗∗∗^*P* < .001.

**Figure 7:** The relationship between RPL4P4 expression and immune checkpoints, TMB, and MSI. (a and b) Correlation analysis between RPL4P4 expression and 47 immune checkpoint genes in cancer. (c) Correlation analysis between RPL4P4 expression and TMB. (d) Correlation analysis between RPL4P4 expression and MSI.

**Figure 8:** RPL4P4 depletion inhibits GBM cell proliferation and migration. (a) Optimal lentivirus was screened using a puromycin kill curve for the stability of the three sets of RPL4P4 lentivirus constructs. (b and c) RPL4P4 knockdown significantly inhibited A-172 and U-251 cell proliferation, as examined by CCK8 assay. (d and i) RPL4P4 knockdown significantly inhibited A-172 and U-251 cell migration as examined by wound healing and Transwell assays. ^∗^*P* < .05, ^∗∗^*P* < .01, and ^∗∗∗^*P* < .001.

**Table 1:** The correlation between RPL4P4 and clinicopathological characteristic in TCGA-glioma dataset.

Characteristic	Low expression of RPL4P4	High expression of RPL4P4	*P*
*n*	348	348	
WHO grade, *n* (%)			**<**0.001
G2	144 (22.7%)	80 (12.6%)	
G3	166 (26.1%)	77 (12.1%)	
G4	0 (0%)	168 (26.5%)	
IDH status, *n* (%)			<0.001
WT	92 (13.4%)	154 (22.4%)	
Mut	255 (37.2%)	185 (27%)	
1p/19q codeletion, *n* (%)			0.842
Codel	88 (12.8%)	83 (12%)	
Noncodel	260 (37.7%)	258 (37.4%)	
Primary therapy outcome, *n* (%)			0.142
PD	77 (16.7%)	35 (7.6%)	
SD	95 (20.6%)	52 (11.3%)	
PR	44 (9.5%)	20 (4.3%)	
CR	78 (16.9%)	61 (13.2%)	
Histological type, *n* (%)			<0.001
Astrocytoma	139 (20%)	56 (8%)	
Glioblastoma	0 (0%)	168 (24.1%)	
Oligoastrocytoma	83 (11.9%)	51 (7.3%)	
Oligodendroglioma	126 (18.1%)	73 (10.5%)	
Age, n (%)			<0.001
≤60	300 (43.1%)	253 (36.4%)	
>60	48 (6.9%)	95 (13.6%)	

**Table 2:** Univariate regression and multivariate survival model of OS in patients with glioma.

Characteristics	Total (*N*)	Univariate analysis		Multivariate analysis	
		Hazard ratio (95% CI)	*P* value	Hazard ratio (95% CI)	*P* value
WHO grade	634				
G2	223				
G3	243	2.999 (2.007-4.480)	<0.001	1.815 (1.077-3.061)	0.025
G4	168	18.615 (12.460-27.812)	<0.001	3.759 (0.961-14.706)	0.057
1p/19q codeletion	688				
Codel	170				
Noncodel	518	4.428 (2.885-6.799)	<0.001	1.244 (0.589-2.624)	0.567
Primary therapy outcome	259				
SD	147				
PD	112	2.288 (1.529-3.426)	<0.001	3.508 (2.049-6.006)	<0.001
SALL4	695				
Low	348				
High	347	1.900 (1.490-2.423)	<0.001	2.275 (1.425-3.633)	<0.001
IDH status	685				
Mut	439				
WT	246	8.551 (6.558-11.150)	**<**0.001	1.600 (0.814-3.145)	0.173
Age	695				
>60	143				
≤60	552	0.214 (0.165-0.278)	**<**0.001	0.247 (0.141-0.430)	<0.001
Histological type	695				
Astrocytoma	195				
Oligoastrocytoma	134	0.657 (0.419-1.031)	0.068	1.186 (0.660-2.129)	0.568
Oligodendroglioma	198	0.580 (0.395-0.853)	0.006	0.565 (0.304-1.051)	0.071
Glioblastoma	168	6.791 (4.932-9.352)	<0.001		
Gender	695				
Female	297				
Male	398	1.262 (0.988-1.610)	0.062	1.583 (0.982-2.554)	0.060

## Data Availability

The data used to support the findings of this study are included within the article and supplementary information file(s).

## Supplementary Materials

Supplementary 1 Supplemental Figure 1: the forest plot showed that in 33 cancers, RPL4P4 had a significant effect on the survival time according to specific tumor types, and RPL4P4 had a clear correlation with prognosis in patients with gliomas (*P* < 0.001).

Supplementary 2 Supplemental Table 1: the correlation between RPL4P4 and clinicopathological characteristic in CCGA-glioma dataset.

Supplementary 3 Supplemental Table 2: univariate regression and multivariate survival model of DFS in patients with glioma.

Supplementary 4 Supplemental Table 3: univariate regression and multivariate survival model of PFS in patients with glioma.
